# Tumor-infiltrating immune cell subpopulations influence the oncologic outcome after intravesical Bacillus Calmette-Guérin therapy in bladder cancer

**DOI:** 10.18632/oncotarget.9537

**Published:** 2016-05-21

**Authors:** Renate Pichler, Josef Fritz, Claudia Zavadil, Georg Schäfer, Zoran Culig, Andrea Brunner

**Affiliations:** ^1^ Department of Urology, Division of Experimental Urology, Medical University of Innsbruck, A-6020 Innsbruck, Austria; ^2^ Department of Medical Statistics, Informatics and Health Economics, Medical University of Innsbruck, A-6020 Innsbruck, Austria; ^3^ Department of Pathology, Division of General Pathology, Medical University of Innsbruck, A-6020 Innsbruck, Austria

**Keywords:** lymphocytes, tumor-associated macrophages, BCG immunotherapy, bladder cancer, tumor microenvironment

## Abstract

Although Bacillus Calmette-Guérin (BCG) is the most successful immunotherapy for high-risk non-muscle-invasive bladder cancer, approximately 30% of patients are unresponsive to treatment. New biomarkers are important to identify patients who will benefit most from BCG during a worldwide BCG shortage. Local immune cell subsets were measured on formalin-fixed, paraffin-embedded tissue sections of bladder cancer by immunohistochemistry, using monoclonal antibodies to tumor-associated macrophages (TAMs; CD68, CD163), B-lymphocytes (CD20) and T-lymphocyte subsets (CD3, CD4, CD8, GATA3, T-bet, FOXP3 and CD25). Cell densities in the lamina propria without invasion, at the invasive front if present, in the papillary tumor stroma, and in the neoplastic urothelium were calculated. Twenty-nine (72.5%) of 40 patients were classified as BCG responders after a mean follow-up of 35.3 months. A statistically significant association was observed for BCG failure with low density of CD4+ and GATA3+ T-cells, and increased expression of FOXP3+ and CD25+ regulatory T-cells (Tregs) as well as CD68+ and CD163+ TAMs. Survival analysis demonstrated prolonged recurrence-free survival (RFS) in patients with an increased count of CD4+ and GATA3+ T-cells. TAMs, Tregs and T-bet+ T-cells were inversely correlated with RFS. Thus, the tumor microenvironment seems to influence the therapeutic response to BCG, permitting an individualized treatment.

## INTRODUCTION

Bacillus Calmette-Guérin (BCG), a live attenuated strain of Mycobacterium bovis, was first introduced in 1921 as a vaccine against tuberculosis [1]. In the 1970′s *Morales et al.* confirmed the efficacy of BCG in bladder cancer [2]. According to the European Association of Urology (EAU) guidelines, BCG immunotherapy still is the most successful adjuvant treatment for high-risk non-muscle-invasive bladder cancer (NMIBC) [3]. However, approximately a third of patients with high-grade recurrence after BCG therapy who underwent consecutive radical cystectomy (RC) were understaged (stage ≥ pT2) [4]; a time delay in RC appears to have been responsible for their reduced disease-specific survival and poor oncologic outcome [4–5] compared to those in whom RC was performed at the time of pathological NMIBC [6]. In times of a worldwide BCG shortage calling for adjustments in the management of bladder cancer [7], novel biomarkers are needed to identify those patients who will benefit from bladder preservation.

BCG-fibronectin complexes were internalized through the tumor resection site. Antigen-presenting cells in the urothelium can phagocytize BCG, which is followed by the presentation of antigen to BCG-specific CD4+ T-cells. Pro-inflammatory cytokines such as IL-1, IL-2, IL-6, IL-8, IL-12, TNF-a and IFN-γ are released, resulting in a predominant Th1-cell-induced immunity with an enhanced recognition of cancer cells through activated macrophages, CD8+ T-cells, natural killer cells and other effector cells [8–9]. Figure 1 shows a schematic overview of BCG-triggered antitumor activity.

**Figure 1:** Schematic view of BCG-induced antitumor activity and important cellular markers After intravesical BCG instillation, BCG molecules can bind to fibronectin through the fibronectin attachment protein (FAP) building BCG-fibronectin complexes. BCG-fibronectin complexes are internalized by urothelial cells and bladder cancer cells at cancer resection sites after surgery. BCG-primed CD4+ T-cells help B-cells to produce antibodies, recruit and activate cytotoxic CD8+ T-cells, macrophages, neutrophils, eosinophils, basophils and natural killer cells, and finally activate DCs that present antigens to CD8+ T-cells. While Th2 type cytokines (IL-4, IL-5, IL-10) have an inhibitory effect on BCG response, activation of a Th1-type immune response through inflammatory cytokines such as IL-1, IL-2, IL-6, IL-8, IL-12, TNF-a and IFN-γ is required for effective BCG-induced antitumor activity.

The immunohistochemical pattern of T-lymphocytes within the tumor microenvironment as well as serum cytokine levels in bladder cancer patients confirmed an imbalance of the Th1/Th2 ratio [10–12]. In therapy-naive bladder cancer patients, BCG immunotherapy may shift the Th2 environment in favor of the Th1-type immune response required for effective BCG-induced antitumor activity and subsequent BCG response [10, 13]. Several trials confirmed a significant increase of Th1-induced urinary cytokines during treatment with intravesical BCG [14–16]. Moreover, pre-therapy levels of Th1/Th2 and tumor-associated macrophage (TAM) polarization of the tumor microenvironment appear to influence BCG response [17–18].

The aim of this pilot study was to determine whether the local density of lymphocyte subpopulations and tumor-associated macrophages (TAMs) in cancer tissue prior to treatment influences recurrence-free survival (RFS) after intravesical BCG therapy.

## RESULTS

### Baseline characteristics

Forty adults aged on average 69 years (SD ± 10.2, range 36–86 years) were included in the study. All patients were treated for primary high-risk NMIBC with adjuvant BCG induction and maintenance therapy. No serious BCG side effects were encountered. Histology confirmed primary CIS, pTa and pT1 urothelial carcinoma in 10 (25.0%), 9 (22.5%) and 21 (52.5%) patients, respectively. Concurrent CIS at the second TURB was confirmed in seven of 30 patients prior to BCG therapy. Seven (17.9%) and 33 (82.1%) were classified as low-grade and high-grade cancers, respectively. Grade 1, 2 and 3 were identified in two (5.0%), nine (22.5%) and 29 (72.5%) tumors. The mean duration of follow-up was 35.3 months (SD ± 22.2, median 29.5 months). Tumor progression with relapse at tumor stage T2 or higher was not observed in any patient. Eleven (27.5%) patients experienced high-grade recurrence after a mean follow-up of 13.8 months while 29 (72.5%) patients were classified as BCG responders. BCG-refractory CIS, T1 high-grade and Ta high-grade were histologically confirmed in three, seven and one patient, respectively. Eight of 11 (72.7%) patients who were BCG failures underwent consecutive RC while three of them refused RC and were treated with 10 cyles of intravesical mitomycin C (MMC) hyperthermia. Three of 11 patients who were BCG failures died of cancer during a mean follow-up of 9.6 months after established BCG failure. No association was found between BCG response and baseline parameters such as age, tumor stage, tumor grade and concurrent CIS (Table 1).

**Table 1:** Univariate Cox proportional hazards models evaluating the association between baseline characteristics, local imune cell subset density in the tumor microenvironment, and BCG failure

Predictors		Univariate		
		HR	95% CI	*P* value
**Gender**	Men	1.00	0.17–3.64	0.755
	Women	0.78		
**Age**	< 70 y	1.00	0.41–4.41	0.629
	≥ 70 y	1.34		
**Stage**	pTa	1.00	0.19–3.04	0.691
	pT1	0.75	0.08–2.80	0.402
	CIS	0.46		
**Grading**	low-grade	1.00	0.29–17.82	0.435
	high-grade	2.27		
**Concurrent CIS**	No	1.00	0.44–6.39	0.446
	Yes	1.68		
CD3^*^		0.52	0.22–1.22	0.135
CD4^*^		0.13	0.02–0.77	**0.025**
CD8^*^		1.02	0.60–1.73	0.944
CD4/CD8 ratio^*^		0.03	0.01–0.23	**0.001**
CD20^*^		1.22	0.67–2.24	0.514
CD68^*^		3.34	2.01–5.55	**< 0.001**
CD163^*^		2.01	1.46–2.77	**< 0.001**
CD163/CD68 ratio^*^		2.38	1.60– 3.53	**< 0.001**
FOXP3^*^		6.05	2.86–12.80	**< 0.001**
CD25^*^		4.27	2.10–8.67	**< 0.001**
GATA3^*^		0.00	0.00–0.09	**0.003**
T-bet^*^		1.54	0.98–2.43	0.062
GATA3/T-bet ratio^*^		0.00	0.00–0.28	**0.017**

* Cox regression with continuous covariate; Hazard ratios are given per one standard deviation increase.

### Pattern of immune cell infiltration in the tumor microenvironment

Significant differences in the localization pattern of immune cell density between the four tumor regions were confirmed for CD3+ (*p* = 0.002), CD4+ (*p* = 0.015), CD8+ (*p* = 0.006), CD20+ (*p* = 0.007), CD25+ (*p* = 0.008) and CD68+ (*p* = 0.010) cells by Friedman two-way ANOVAs. Immune cell infiltration was significantly increased in the lamina propria without invasion compared to the neoplastic urothelium for CD3 (*p* = 0.001), CD4 (*p* = 0.010), CD8 (*p* = 0.004), CD20 (*p* = 0.006), CD25 (*p* = 0.011) and CD68 (*p* = 0.012), Figure 2.

**Figure 2:** Total expression levels of immune cell subsets stratified by tumor region (A–J) Lamina propria without invasion (LP) *vs.* tumor stroma (TS) *vs.* neoplastic urothelium (NU) *vs.* invasive front (IF). Black lines represent the mean (*p < 0.05; **p < 0.01; ***p < 0.001; Friedman's two-way ANOVAs and Wilcoxon's signed-rank tests).

### Gender-specific differences

The male to female ratio of the study population was 4:1 (32 men *vs.* 8 women). Gender was not associated with BCG failure (hazard ratio [HR] = 0.78; 95% CI 0.17–3.64; *p* = 0.755), Table 1. Furthermore, no sex-specific difference was observed in the total number of immune cell subsets. The mean expression level of each tumor-infiltrating immune cell subset was similar in women and men [727.7 *vs.* 781.7 (CD3+); 353.2 *vs.* 392.2 (CD4+); 216.2 *vs.* 284.4 (CD8+); 82.6 *vs.* 144.1 (CD20+); 157.5 *vs.* 156.6 (CD68+); 150.7 *vs.* 166.6 (CD163+); 44.2 *vs.* 50.8 (FOXP3+); 53.2 vs. 70.9 (CD25+); 268.7 *vs.* 304.9 (GATA3+) and 62.1 *vs.* 91.2 (T-bet+)]. In addition, gender had no significant effect on RFS (*p* = 0.753), Figure 3.

**Figure 3:** Influence of gender on total expression levels of immune cell subsets (A–D) and recurrence-free survival (E) Data represent mean ± SEM; Mann-Whitney *U* test.

### Correlation analysis of immune cell subsets

Several associations were observed between the infiltration density of CD3 and CD8 (*r*_s_ = 0.90, *p* < 0.001), CD3 and CD4 (*r*_s_ = 0.92, *p* < 0.001), CD3 and GATA3 (*r*_s_ = 0.73, *p* < 0.001), CD3 and T-bet (*r*_s_ = 0.66, *p* < 0.001), and between CD3 and CD20 (*r*_s_ = 0.51, *p* = 0.014). In addition, FOXP3 was correlated with CD25 (*r*_s_ = 0.79, *p* < 0.001), CD68 (*r*_s_ = 0.75, *p* < 0.001) and CD163 (*r*_s_ = 0.69, *p* < 0.001). A significant correlation between CD68 and CD163 (*r*_s_ = 0.89, *p* < 0.001) was identified, whereas CD25 (*r*_s_ = −0.57, *p* = 0.002), FOXP3 (*r*_s_ = −0.62, *p* < 0.001), CD163 (*r*_s_ = −0.63, *p* < 0.001) and CD68 (*r*_s_ = −0.66, *p* < 0.001) were inversely correlated with the CD4/CD8 ratio. Moreover, TAMs were negatively correlated with CD3+, CD4+ and CD8+ T-cells, but without statistical significance.

### Density of local immune cell subsets and histopathological parameters

With regard to CD3+, CD4+ and CD8+ T-cells, CD20+ B-cells, CD25 and FOXP3+ Tregs as well as GATA3+ and T-bet+ T-cell infiltration, CD4/CD8, CD163/68 and GATA3/T-bet ratio, no association was registered between total counts and tumor grade. However, pT1 bladder cancers confirmed the highest count (mean ± SD) of CD3+ T cells (983.7 ± 662.0; *p* = 0.022), CD8+ T cells (359.9 ± 238.0; *p* = 0.008) and CD68+ TAMs (181.6 ± 93.9; *p* = 0.014) compared to pTa bladder cancer and CIS. In contrast, CD20+, CD4+, CD25+, FOXP3+, CD163+, T-bet+ and GATA3+ cell density as well as CD4/CD8, CD163/68 and GATA3/T-bet ratio did not differ significantly between the different tumor stages, Figure 4.

**Figure 4:** Total expression levels of immune cell subsets depending on BCG response (A–D), tumor grade (E–H) and tumor stage (I–L) Data represent mean ± SEM (*p < 0.05; **p < 0.01; ***p < 0.001; Mann-Whithney *U* test and independent-samples Kruskal-Wallis test).

### Tumor-infiltrating lymphocyte subsets and BCG outcome

Significant differences in mean expression levels based on BCG response were confirmed for CD4+ T-cells (failure *vs.* response: 161.2 *vs.* 469.0; *p* = 0.002), GATA3+ T-cells (44.9 *vs.* 393.6; *p* < 0.001) and T-bet+ T-cells (123.7 *vs.* 70.8; *p* = 0.033). In addition, the CD4/CD8 ratio (mean ± SD, 2.01 ± 0.75 *vs.* 0.54 ± 0.15; *p* < 0.001) and the GATA3/T-bet ratio (7.17 ± 4.75 vs. 0.41 ± 0.16; *p* < 0.001) were significantly increased in BCG responders compared to BCG failures. In contrast, levels of CD3+ (*p* = 0.229), CD8+ (*p* = 0.437) T-cells and CD20+ (*p* = 0.952) B-cells did not differ significantly in regard of the oncologic outcome, Figure 4.

CD4+ T-cell count [HR = 0.13; 95% CI: 0.02–0.77; *p* = 0.025], CD4/CD8 ratio [HR = 0.03; 95% CI: 0.01–0.23; *p* = 0.001], GATA3+ T-cells [HR = 0.00; 95% CI: 0.00–0.09; *p* = 0.003] and GATA3/T-bet ratio [HR = 0.00; 95% CI: 0.00–0.28; *p* = 0.017] were associated with failed BCG therapy, Table 1. Moreover, ROC analysis revealed that the total CD4+ T-cell density (AUC=0.80; 95% CI: 0.65−0.91; *p* = 0.003), total T-bet+ T-cell density (AUC = 0.72; 95% CI: 0.56–0.85; *p* = 0.033) and total GATA3+ T-cell density (AUC = 0.99; 95% CI: 0.89–1.00; *p* < 0.001) were able to predict BCG failure.

The local (mean ± SD) expression of CD25+ (117.6 ± 34.9) and FOXP3+ Tregs (111.0 ± 23.6) was significantly higher in patients with BCG failure compared to BCG responders (48.3 ± 36.5; *p* < 0.001 for CD25 and 26.2 ± 13.8; *p* < 0.001 for FOXP3), Figure 4.

Univariate analysis confirmed a significant positive association between CD25+ [HR = 4.27; 95% CI: 2.10−8.67; *p* < 0.001], FOXP3+ Tregs [HR = 6.05; 95% CI: 2.86–12.80; *p* < 0.001] and BCG failure, Table 1. Significantly better prediction of BCG failure was confirmed by total CD25+ cell density (AUC = 0.92; 95% CI: 0.79–0.98; *p* < 0.001) and total FOXP3+ cell density (AUC = 1.00; 95% CI: 0.91–1.00; *p* < 0.001) on ROC analysis.

### CD68+ and CD163+ tumor associated macrophages (TAMs) and BCG outcome

The median number of total CD68+ and CD163+ TAMs was significantly increased in patients with BCG failure compared to BCG responders (290.4 and 386.5 *vs.* 106.2 and 78.9; *p* < 0.001). Similarly, we observed a significantly higher CD163/CD68 ratio (mean ± SD) in patients with recurrence (1.32 ± 0.23) than in patients with BCG response (0.73 ± 0.19; *p* < 0.001), Figure 4.

Univariate Cox regression analysis revealed that tumors presenting high number of CD68+ TAMs [HR = 3.34; 95% CI: 2.01–5.55; *p* < 0.001], high numbers of CD163+ TAMs [HR = 2.01; 95% CI: 1.46–2.77; *p* < 0.001] and a high CD163/CD68 ratio [HR = 2.38; 95% CI: 1.60–3.53; *p* < 0.001] were associated with a greater risk of recurrence after BCG therapy, Table 1.

Moreover, significantly better prediction of BCG failure was confirmed by total CD68+ TAM density (AUC = 1.00; 95% CI: 0.91–1.00; *p* < 0.001) and by CD163+ TAM density (AUC = 1.00; 95% CI: 0.91–1.00; *p* < 0.001) on ROC analysis.

### Influence of immune cell subset expression on RFS after BCG therapy

Finally, we investigated the relationship between the infiltration level of immune cell subsets in the pretreatment microenvironment and RFS. Patients were divided into two groups (low *vs.* high count), based on the median count of each immune cell subtype for survival analysis (median cell density: 579.5 for CD3; 238.0 for CD4; 241.0 for CD8; 1.48 for CD4/CD8 ratio; 84.5 for CD20; 129.5 for CD68; 96.0 for CD163; 0.85 for CD163/CD68 ratio; 33.0 for FOXP3; 63.0 for CD25; 180.5 for GATA3, 71.0 for T-bet, and 4.3 for GATA3/T-bet ratio). An increased count of CD4+ T-cells and GATA3+ T-cells was associated with a significantly prolonged RFS compared to patients with a low CD4+ T-cell count (mean, 83.8 *vs.* 37.4 months, *p* = 0.013) or a low GATA3+ T-cell count (*p* = 0.002). In contrast, RFS was significantly lower in patients with high numbers of T-bet+ T-cells (*p* = 0.009), CD68+ TAMs (*p* < 0.001), CD163+ TAMs (*p* < 0.001), CD25+ (*p* = 0.003) and FOXP3+ Tregs (*p* < 0.001) than in patients with low counts, Figure 5. The density of CD3+ (*p* = 0.388), CD8+ (*p* = 0.229) T-cells and CD20+ B-cells (*p* = 0.718) did not signicantly predict RFS.

**Figure 5:** Kaplan-Meier survival curves Recurrence-free survival (RFS) in months according to total CD4+, T-bet+, GATA3+, CD25+, FOXP3+, CD68+ and CD163+ cell count stratified by the predefined cutoff points (≤ median = low count; > median = high count). *P* values by log-rank test; *p < 0.05; **p < 0.01; ***p < 0.001.

## DISCUSSION

Despite the introduction of BCG for bladder cancer treatment in 1976 [2], no reproducible biomarkers are available in clinical practice for predicting BCG response. However, urinary IL-2 levels are currently the most promising markers in predicting BCG response [19]. A signature of nine urinary cytokines including TNF-alpha, IL-2, IL-8, IL-6, IL-1ra, IL-10, IL-12[p70], IL-12[p40] and TRAIL showed an accuracy of 85.5% in predicting recurrence after BCG [20].

Tumor-infiltrating immune cells influence cancer-specific survival in bladder cancers with either poor or improved prognosis, depending on their subsets and polarization. A low T effector/Treg cell ratio was associated with early recurrence [21]. In muscle-invasive bladder cancer, patients with FOXP3 expression in tumor cells had reduced long-term survival compared to patients with FOXP3-negative cancers [22]. Horn *et al.* (2015) showed that a high FOXP3/CD8 ratio within invasive cancer tissue was an independent predictor of poor overall survival after cystectomy [23]. High numbers of CD68+ TAMs were associated with an advanced pT category and high-grade cancer [24], acting as an additional independent factor (CD68/CD3 ratio > 1) with a more than 7-fold higher risk of cancer-specific death on multivariate analysis [25]. Conversely, increased intratumoral CD3+ and CD8+ T-cells were predictive of significantly better overall and disease-free survival [26–27].

The tumor microenvironment can regulate therapeutic resistance. Nevertheless, the potential influence of tumor-infiltrating lymphocyte subpopulations in the tumor microenvironment on BCG response in bladder cancer has not been clarified yet. The induction of urinary and serum Th1 cytokines is a common feature in BCG responders [10, 13−16, 28]. Luo *et al.* (2003) identified additional costimulatory cytokines in humans (IL-2 and IL-12) and *in vivo* (IL-18 and IL-12), which increase BCG antitumor activity by greater IFN-γ production compared to BCG alone [29]. Moreover, patients with a preexisting BCG immunity experienced a significant improvement in recurrence-free survival. This phenomenon may be explained by the fact that parenteral exposure to BCG prior to therapy triggers accelerated T cell infiltration into the bladder wall compared to standard BCG treatment [30]. Honda *et al.* (1997) noticed, in a small number of 16 patients, a significant increase of CD3+, CD4+ and CD8+ T-cells in tissue specimens after adjuvant BCG therapy. Although BCG responders tended to show higher T-cell infiltration levels compared to BCG failure, the differences were not statistically significant [31]. Our results show that an increased intratumoral CD4+ T-cell population was significantly associated with BCG response (Figure 4A) and longer RFS (Figure 5A). Interestingly, a preexisting Th1 tumor microenvironment in patients with primary CIS was predictive of BCG failure in a study by Nunez-Nateras *et al.* [17]. The authors hypothesized that adding BCG to activate intratumoral Th1 immune response is unlikely to increase a Th1-activated cancer microenvironment [17]. Our results are in line with the observations made by Nunez-Nateras *et al.* [17]. We registered a positive association between an increased GATA3/T-bet ratio and a prolonged recurrence-free survival. Furthermore, the total T-bet+ T-cell counts in BCG responders were significantly lower than those of patients with BCG failure. However, the influence of Th1/Th2 polarization in the tumor microenvironment on BCG response has not been validated in large studies. Both Th1 and Th2 genes increased in the bladder of tumor-bearing mice after cancer cell implantation. However, the Th1/Th2 balance changed depending on the time after bladder cancerogenesis; while GATA3 decreased at day 7, T effector cells significantly increased at day 28 [32]. Therapeutic strategies with a bimodal function inducing a Th1 response and blocking a pre-therapeutic Th2 milieu in Th2-dominated tumors have shown to improve responses to immunotherapy [32–33]. Also BCG is thought to be a Th1-polarized immunomodulator [34]. In our study, BCG responders noticed a predominant Th2 tumor microenvironment with high levels of GATA3+ T-cells and increased GATA3/T-bet ratio. To confirm the shift in favor of a Th1-type microenvironment in responders, post-BCG tumor tissue analysis would be necessary for comparison. As BCG response has not been verified by biopsy, no post-therapy tumor tissue is available for comparative analysis.

Tumor-infiltrating Tregs are key players in the tumor immune escape mechanism, inhibiting the antitumor response in various cancer entities [35–38] with a poor oncologic outcome. An increased frequency of intratumoral FOXP3+ Tregs and inhibitory cytokines such as IL-10 and TGF-β was noted in bladder cancer patients compared to the healthy population [12, 22–23, 39]. Interestingly, Treg frequencies and CD25^high^ and FOXP3- cells in peripheral blood were similar in different patient groups (control group, localized BCa, lymphogen metastatic BCa and distant metastatic BCa). CD25high and FOXP3- cell populations were significantly reduced after surgery while chemotherapy with gemcitabine/cisplatin had no effect [40]. Another trial showed that a low CD4+CD25+FOXP3+ Treg frequency after radical cystectomy in pT2-pT4 tumors was associated with poor survival. The authors think that this post-surgery Treg decrease may indicate a tumor-specific immune tolerance during tumor advancement [41]. Moreover, Tregs can suppress effector mechansims of the immune response in a variety of vaccination models [42–44]. Quinn *et al.* (2008) analyzed the effect of Treg inactivation prior to BCG vaccination on the development of protective immunity in a murine model. Although Treg inactivation increased the number of IL-2 or IFN-γ-producing CD4+ lymphocytes, the presence of CD4+CD25+ Tregs during vaccination did not significantly influence the protective efficacy of the BCG vaccine [45]. However, a simultaneous inhibition of Th2 cells and Tregs appears to enhance host-protective immunity [46] and BCG-induced vaccine efficacy in BCG-vaccinated mice [47], thus inducing increased Th1 response. The present study revealed, for the first time, that a high density of CD25+ (HR = 4.27) and FOXP3+ (HR = 6.05) T-cells in the tumor microenvironment was predictive of BCG failure.

TAMs are also an important element of the so-called tumor stroma. TAMs are markedly present in many cancer entities [48–49], promoting neoangiogenesis, the production of immunoregulatory, immunosuppressive molecules and growth factors, eventually culminating in tumor progression and reduced cancer-specific survival [50]. The infiltration levels of TAMs in relation to the efficacy of BCG immunotherapy have been investigated most intensively. Several studies confirmed that a large number of TAMs infiltrating cancer cells and an increased cancer cell-to-lamina propria TAM ratio were associated with a poor oncologic outcome after BCG [18, 51–52]. Interestingly, the strongest TAM infiltration was registered in the stroma. We also observed the strongest CD68+ and CD163+ TAM infiltration in the tumor stroma and lamina propria. An increased density of M2-polarized macrophages in the stroma, but not in tumor cells, was related to BCG failure and a 2.6-fold higher risk of recurrence [52–53]. Conversely, CD68+ TAMs in stroma or within tumor nests were found to have no effect on the outcome of BCG [54]. In the present study, total levels of CD163+ (HR = 2.01, *p* < 0.001) and CD68+ TAMs (HR = 3.34, *p* < 0.001) were associated with reduced BCG response. We observed a significant correlation between T-, and B-lymphocyte marker scores, TAM and Treg cell marker scores in the tumor microenvironment, suggesting that the immunological response to BCG is a complex mechanism involving more than one specific immune cell subpopulation [25].

One of the major limitations of the present pilot study is the heterogeneous and retrospective character of the limited patient number, including tumors with and without superficial invasion (pTa and pT1) as well as carcinoma *in situ* (CIS). Multivariate analysis was not performed because of the small sample size and multicollinearity. Thus, no statement can be made about independent predictors of BCG response. However, the presented findings are clearly hypothesis generating. Furthermore, tumor tissue analysis was performed by immunohistochemistry (IHC) with possible bias (antigen retrieval, detection system, specimen fixation, antibody panel selection, interpretation of IHC expression) that may influence the analysis of IHC reactions. Moreover, IHC enables quantitative but not functional analysis. Prospective urinary and serum cytokine measurements or flow cytometry analysis during BCG instillations would be helpful to gain further knowledge about the systemic BCG-induced immune response.

## CONCLUSIONS

We showed that increased pretreatment levels of tumor-infiltrating Tregs and TAMs, and a decreased density of Th2-predominant CD4+ T-cells contribute to poor recurrence-free survival after BCG therapy. New pretreatment biomarkers will help to identify patients who are more like to benefit from bladder preservation strategy in times of a worldwide BCG shortage. However, these findings must be re-evaluated in further prospective trials with sufficient statistical power prior to draw any final conclusion. Prognostic models would be helpful to prove the clinical applicability of those immune cell markers within the tumor microenvironment.

## MATERIALS AND METHODS

### Patients and clinical characteristics

After approval by the local ethics committee (study number AN2014-0121; 336/4.3), medical records of patients with primary, high-risk NMIBC undergoing consecutive intravesical BCG therapy after transurethral resection of the bladder (TURB) were reviewed retrospectively. A second TURB within 2–6 weeks after initial resection was performed in all patients (except carcinoma *in situ*) to exclude residual tumor or understaging. According to the EAU guidelines [3], intravesical BCG induction therapy was given in a 6-weekly schedule once a week, followed by maintenance therapy for 1–3 years (3-weekly once a week at 3, 6, 9, 12, 18, 24, 30 and 36 months). Each intravesical instillation through a sterile disposable catheter contained 2 × 10^8^ to 3 × 10^9^ viable units from live attenuated strain of BCG bacteria seed RIVM derived from seed 1173-P2 (BCG Medac, Wedel, Germany). Each solution was retained for 1 to 2 hours. Oncologic follow-up was performed with cystoscopy and urinary (voided urine and bladder washing) cytology every 3 months for a period of 2 years, then every 6 months for 5 years, and once every year thereafter [3], at our oncological outpatient department. Upper urinary tract imaging with computed tomography urography was performed initially at the time of diagnosis, and repeated once a year or in case of tumor recurrence. In case of disease recurrence, the tumor was resected transurethrally. A muscle-invasive bladder cancer detected during follow-up (progression) or a high-grade relapse (recurrence) after BCG therapy was interpreted as BCG failure. Recurrence-free survival (RFS) was defined as the time from the date of surgery to tumor recurrence, or the last oncologic follow-up when no relapse occurred.

### Tumor samples

All patients gave their written informed consent to perform further analysis on tumor samples obtained at the time of surgery. All tumor specimens after TURB were reviewed in regard of diagnosis, tumor grade (WHO 1973 and 2004) and stage (TNM 2009) by two uropathologists with long-standing experience (A.B. and G.S.). One representative tumor block of every case was selected for further immunohistochemical analysis. Consecutive slides were used to compare the same field of view in a given case. Our study cohort included tumors with and without superficial invasion (Ta and T1) as well as carcinoma *in situ* (CIS). Therefore, the localization patterns of tumor-infiltrating immune cells were analyzed in four different regions: in the lamina propria without invasion, at the invasive front if present, in the papillary tumor stroma if present, and in the neoplastic urothelium, Figure 6. In case of CIS, only the underlying lamina propria without invasion and the overlying neoplastic urothelium were used for analysis.

**Figure 6:** Hematoxylin and eosin staining for representative images of analyzed tumor areas (**A**) Exophytic papillary non-invasive bladder cancer with scarce inflammation of the underlying lamina propria (scale bar: ~100 μm); (**B**) invasive front of a pT1 bladder cancer with dense lymphocytic infiltration around invasive tumor cell nests (scale bar: ~40 μm); (**C**) superficial tumor papillae with discrete lymphocytic infiltration of papillary stroma and neoplastic urothelial cells (scale bar: ~40 μm); (**D**) CIS with widened vessels and inflammation of the underlying lamina propria (scale bar: ~40 μm).

### Immunohistochemistry (IHC)

A panel of 10 primary antibodies was used for subtyping the inflammatory infiltrate within the tumor microenvironment. T-cells were labeled using a CD3 antibody (Monoclonal Rabbit Anti-Human CD3, Clone 2GV6, prediluted, Roche). T-helper cells (Th), type 1 T-helper (Th1) cells, and type 2 T-helper (Th2) cells were assessed with a CD4 antibody (Lyophilized Monoclonal Mouse Anti-CD4, Clone 1F6, dilution 1:10, Leica), a T-bet antibody (Monoclonal Rabbit Anti-Human T-bet, Clone MRQ-46, prediluted, Roche) and a GATA3 antibody (Monoclonal Mouse Anti-Human GATA3, Clone L50-823, prediluted, Roche). Cytotoxic T-cells were labeled by CD8 antibody (Monoclonal Mouse Anti-Human CD8, Clone C8/144B, dilution 1:50, Dako). In addition, regulatory T-cells (Tregs) were examined with a FOXP3 (Monoclonal Mouse Anti-FOXP3, Clone 236A/E7, dilution 1:100, Abcam) and a CD25 antibody (Monoclonal Mouse anti-Human CD25, Clone 4C9, prediluted, Roche). TAMs were labeled using a CD68 antibody (Monoclonal Mouse Anti-Human CD68, Clone PG-M1, dilution 1:50, Dako) for M1 polarization and a CD163 antibody (Monoclonal Mouse anti-Human CD163, Clone MRQ-26, prediluted, Roche) for M2 polarization. Finally, B-lymphocytes were assessed using a CD20 antibody (Monoclonal Mouse Anti-Human CD20, Clone L26, prediluted, Roche). For positive control human tonsil was used for all markers. Neoplastic urothelium served as an additional internal positive control for GATA3. For negative control, slides from human tonsil were incubated without primary antibody. Representative stains and quantifications for CD3, CD4, CD8, FOXP3, CD25, and CD68 and CD163 are shown in Figures 7–9.

**Figure 7:** Immunohistochemistry for CD3+, CD4+, CD8+ T-cells Lamina propria of a high-grade papillary urothelial carcinoma. Representative images of T-cell subsets stained with anti-CD3, anti-CD4 and anti-CD8 (brown). High infiltration of CD3+, CD4+ and CD8+ T-cells (**A**, **C**, **E**) compared to low expression (**B**, **D**, **F**). (**G**) Quantification showing a positive correlation between CD3+ T cells and other effector immune cells (CD4+ and CD8+ T-cells); *r*_s_ = Spearman's rank correlation coefficient; *p*-values for r_s_ were corrected for multiple testing according to the Bonferroni method. Scale bar (A–F): ~40 μm.

**Figure 8:** Immunohistochemistry for regulatory T-cells Regulatory T-cells in a patient with BCG response (**A**, **C**) and BCG failure (**B**, **D**). Representative stains are shown for FOXP3 and CD25. Decreased FOXP3+ and CD25+ T-cell expression in BCG response compared to BCG failure. (**E**) Quantification showing a statistically significant positive correlation between CD25+ and FOXP3+ T-cells; r_s_ = Spearman's rank correlation coefficient; *p*-values for r_s_ were corrected for multiple testing according to the Bonferroni method. Scale bar (A–D): ~40 μm.

**Figure 9:** Immunohistochemistry for tumor-associated macrophages CD68+ and CD163+ macrophage infiltration in a patient with BCG response (**A**, **C**) and BCG failure (**B**, **D**). Representative micrographs showing a low infiltration of CD68+ and CD163+ TAMs in BCG response in comparison to BCG failure. (**E**) The density of CD68+ TAMs was positively correlated with CD163+ TAMs; r_s_ = Spearman's rank correlation coefficient; *p*-values for r_s_ were corrected for multiple testing according to the Bonferroni method. Scale bar (A–D): ~40 μm.

Staining was performed using an automated immunostainer (BenchMark ULTRA, Ventana Medical Systems, Tucson, US). Briefly, formalin-fixed, paraffin-embedded (FFPE) tissue sections were cut in widths of 1.5 μM. After deparaffinization, the slides were treated with cell conditioning reagent 1 (CC1, Ventana Medical Systems, Tucson, US) for antigen retrieval. Primary antibodies were incubated for 32 minutes at 37°C. The Ultra View DAB Detection Kit (Ventana Medical Systems, Tucson, US) was used for visualization, in accordance with the manufacture's recommendation. Finally, slides were washed in distilled water, counterstained with hematoxylin (12 minutes) and bluing reagent (4 minutes), dehydrated in a descending order of alcohols, cleared in xylene, and coverslipped with Tissue-tek mounting medium (Sakura Finetek, Japan).

### Quantification of immune cell density

Systematic quantitative cell analysis was performed by counting manually the number of positive cells for each subset in a maximum of 5 high-power fields (HPF) in each tumor region, using the same field of view in consecutive slides. The number per field, per tumor level and the total count of positive cells in 4 different regions for each subset was quantified. In addition, the CD4/CD8 ratio as well as the Th2/Th1 ratio and CD163/CD68 ratio were assessed. All counts were performed by two independent observers using an Olympus BX50 microscope (40× magnification) equipped with the ProgResC10plus camera (Jenoptik, Jena, Germany). Each investigator was blinded for the BCG outcome and repeated the counts twice. For all immune cell markers excellent intra- and interobserver reliability was achieved (all interobserver ICCs > 0.980; all intraobserver ICCs for examiner 1 > 0.985 and > 0.960 for examiner 2). Thus, the average of all four counts was used for further statistical analysis.

### Statistics

Baseline characteristics and infiltration levels of immune cell subsets were compared with Fisher's exact tests and (due to skewed distributions of most parameters) Mann-Whitney U tests and independent Kruskal-Wallis tests, based on gender, tumor grade, tumor stage and BCG response status. To assess reliability of assessments, intra- and interclass correlation coefficients (ICC) for two-way mixed measures (single measures for intra-, and average measures for interobserver variability) were calculated. Friedman's two-way analysis of variance (ANOVA) and Wilcoxon's signed-rank tests were used for comparison of paired groups (tumor regions). Correlations between parameters were assessed with Spearman's ρ correlation coefficient (*r*_s_). The predictive power of all marker expression levels on BCG response was evaluated by plotting receiver operating characteristic (ROC) curves and calculating the area under the curve (AUC) with exact binomial 95% confidence intervals (95% CI). Univariate Cox proportional hazards models were used to estimate hazard ratios (given per one standard deviation increase) and 95% CIs for BCG failure. Since multivariate analyses revealed numerically unstable results due to small sample size and multicollinearity, the results are not mentioned here. The median value of each marker was used as the cutoff point to dichotomize the patients into two groups (low *vs.* high count) for Kaplan-Meier survival analysis and comparison by the log-rank test. A significance level of *α* = 0.05 (two-tailed) was applied for all *p*-values; *p*-values for correlation coefficients were corrected for multiple testing according to the Bonferroni method. SPSS, version 22.0 (SPPS Inc., Chicago, IL, USA) was used for statistical analysis. Graphic diagrams were produced with GraphPad PrismTM6 (GraphPad Software Inc., La Jolla, CA). All values were presented as mean ± standard error of the mean (SEM).
